# One-step Conjugation of Glycyrrhetinic Acid to Cationic Polymers for High-performance Gene Delivery to Cultured Liver Cell

This article has been retracted.

**DOI:** 10.1038/srep21891

**Published:** 2016-02-23

**Authors:** Yue Cong, Bingyang Shi, Yiqing Lu, Shihui Wen, Roger Chung, Dayong Jin

**Affiliations:** 1 Institute of Pharmacy, Pharmaceutical College, Henan University, Jin Ming Avenue, Kaifeng, Henan, 475004, China; 2 College of Life Sciences, Henan University, Jin Ming Avenue, Kaifeng, Henan, 475004, China; 3 Advanced Cytometry Labs, ARC Centre of Excellence for Nanoscale BioPhotonics (CNBP), Macquarie University, Sydney, NSW, 2109, Australia; 4 Faculty of Medicine & Health Sciences, Macquarie University, Sydney, NSW, 2109, Australia

## Abstract

Gene therapies represent a promising therapeutic route for liver cancers, but major challenges remain in the design of safe and efficient gene-targeting delivery systems. For example, cationic polymers show good transfection efficiency as gene carriers, but are hindered by cytotoxicity and non-specific targeting. Here we report a versatile method of one-step conjugation of glycyrrhetinic acid (GA) to reduce cytotoxicity and improve the cultured liver cell -targeting capability of cationic polymers. We have explored a series of cationic polymer derivatives by coupling different ratios of GA to polypropylenimine (PPI) dendrimer. These new gene carriers (GA-PPI dendrimer) were systematically characterized by UV-vis,^1^H NMR titration, electron microscopy, zeta potential, dynamic light-scattering, gel electrophoresis, confocal microscopy and flow cytometry. We demonstrate that GA-PPI dendrimers can efficiently load and protect pDNA, via formation of nanostructured GA-PPI/pDNA polyplexes. With optimal GA substitution degree (6.31%), GA-PPI dendrimers deliver higher liver cell transfection efficiency (43.5% vs 22.3%) and lower cytotoxicity (94.3% vs 62.5%, cell viability) than the commercial bench-mark DNA carrier bPEI (25kDa) with cultured liver model cells (HepG_2_). There results suggest that our new GA-PPI dendrimer are a promising candidate gene carrier for targeted liver cancer therapy.

Liver cancer is the sixth most common cancer in the world and the third most common cause of death from cancer^1^. Gene therapy, delivering a therapeutic nucleic acid into the chromosomes of diseased cells to regulate or replace abnormal genes, is a promising approach for cancer treatment benefiting from the rapid development of knowledge in elucidating the molecular basis of cancer and the complete sequence information of the human genome^2^. The success of gene therapy is now largely dependent upon the development of high-performance delivery systems which can efficiently and selectively deliver therapeutic genes into target cancer cells without causing associated side-effects.

In contrast to viral vectors, non-viral synthetic vectors have good biocompatibility, satisfactory DNA loading capability and can be easily functionalized for improved gene delivery^3^,^4^,^5^. In the last decade, researchers have explored multitudes of synthetic gene carriers for gene therapy^6^,^7^,^8^,^9^. Among the more commonly used synthetic gene vectors such as polyethyleneimine (PEI), dendrimers, polylysine, Polycation, poly(ether ester amide)s, chitosan, and poly(2-(dimethylamino)-ethyl methacrylate), polypropylenimine (PPI) dendrimers have been used as one of the most efficient carriers for gene/drug delivery due to their unique combination of high charge density for high-capacity gene loading, advanced structure for versatile surface modification and amenable intermolecular space for entrapment of host-molecule with excellent proton sponge effect for endosome escape^10^,^11^,^12^,^13^,^14^,^15^,^16^. But the high cytotoxicity and non-specific cell-targeting properties of PPI dendrimers hinder their potential applications in hepatic gene delivery^17^,^18^,^19^.

The high toxicity of PPI is caused mainly by their high positive charge, which can be alleviated by surface modification of PEGlation, Glycolation and carbohydrate-coating^18^. To enhance their targeting capability, these carriers can be intensively functionalized with targeting ligands^20^, such as antibodies^21^,^22^ and sugars^23^, for transporting therapeutic cargos to the liver and the treatment of hepatocellular carcinoma. Recent successes have been achieved for antibody-mediated liver cancer targeting (including using the Licartin^24^), however broad application of these strategies has been limited by the costs associated with antibody production and humanisation. Recently, facile one step preparation (synthesis/conjugation) strategy has been attracted more attentions for the development of advanced functional materials because it is faster, sampler, more efficient and with higher product yields comparing with multi-step fabrication process^25^,^26^. Therefore, how to realize the alleviation of cytotoxicity and enhancement of targeting capability of PPI dendrimer via one step fabrication process is important for the development of PPI dendrimer based advanced delivery systems.

Glycyrrhetinic acid (GA), a type of traditional Chinese medicine which is the main bioactive compounds extracted from licorice^27^,^28^, has been demonstrated as an efficient targeting ligand for liver cells due to the existence of specific GA receptors on the cellular membrane of hepatocytes^29^,^30^,^31^,^32^. Accordingly, growing interest has been focused on the application of GA to modify the gene/drug carriers for liver targeting. To our best knowledge, GA has not been used to functionalize highly cationic polymers such as PPI, which can potentially not only endow the liver cell targeting capability but also minimize the cytotoxicity of cationic polymers via exploring facile one step coupling, towards high-performance gene delivery systems.

This study focuses upon the bio-conjugation of GA onto PPI dendrimers to enhance their liver cell targeting capacity and minimize cytotoxicity. This is achieved through GA-linkage decreasing the positive charge density of PPI dendrimer and specifically mediating endocytosis through GA receptors (Fig. 1). Importantly, we have developed one-step synthesis of GA-PPI dendrimers through introduction of GA to the backbone of the PPI dendrimer backbone by EDC chemistry with fine tuning substitution (Fig. S1, Supporting Information). This provides a series of cationic polymer derivatives possessing different substitution degrees of GA, allowing us to optimize specific chemical and biological functions of GA-PPI dendrimers by upon the influence of the degree of GA modification. DNA binding and protection capability, particle size and zeta potentials, cytotoxicity, and targeted gene delivery capability of GA-PPI carriers were also systematically studied.

## Result and Discussion

### Synthesis and confirmation of GA-PPI conjugation

A series of GA-PPI dendrimer derivatives were developed through conjugation of GA onto the surface of Generation-4 PPI dendrimer via EDC chemistry. Incremental amounts of GA substitution were introduced to produce 8 samples of GA-PPI conjugates by changing the feed ratio of GA to PPI dendrimer (details see Methods). The successful conjugation of GA to PPI dendrimer was evident from UV-vis measurement and the ^1^H-NMR spectrum. From the UV-vis absorption of GA-PPI dendrimers at the wavelength of 250 nm, the GA substitutions degrees on GA-PPI dendrimers ranging from 0.9% to 32.08% were determined (Table S1 and Fig. S2, Supporting Information). The coupling of the GA to PPI dendrimer was further confirmed from the ^1^H-NMR spectrum, where the proton signal of GA (δ 0.5 to 2.0 ppm) and that from PPI dendrimer (δ 2.4 to 3.5 ppm) were both present (Supplementary Fig. S3). Additionally, the water solubility of the dendrimers was assessed by measuring the transmittance of GA-PPI dendrimers under different pH from 6 to 10, which showed that the transmittance decreases with the increase of GA substitution. Nevertheless, except for GA-PPI-8, the transmittance of GA-PPI dendrimers was always above 80%, indicating their excellent water solubility under physiological conditions (Supplementary Fig. S4).

### Self-assembly of GA-PPI/pDNA polyplexes

An ideal cationic dendrimer-based gene carriers should have the capacity to self-assemble the negatively charged cargo-pDNA into polyplex nanoparticles (50–150 nm) that can be up-taken *via* endocytosis. Notably, larger nanoparticles (up to 1 μm) are believed to be preferentially internalised through a slow, non-degradable, caveolae-mediated route^33^. Since the endocytic machinery and cell membrane have well-defined geometries and flexibility that restrict the entry of incompatible particles, the control of polyplex particle size is crucial for gene delivery. In this work, our GA-PPI dendrimers were mixed with naked pDNA (as the DNA cargo) at different charge (N/P) ratios of carrier to pDNA (details see methods section). In the presence of negatively charged pDNA, cationic GA-PPI dendrimers can self-assemble into nanosized GA-PPI/pDNA polyplexes, similar in size to the original PPI dendrimers. As shown in Fig. 2A, the apparent particle size of the (GA-) PPI/pDNA polyplexes measured by dynamic light scattering (DLS) decreases from a few micrometres to 100 nanometres as the N/P ratio increases from 0.5 to 30 in all cases. At a fixed N/P ratio, the GA-PPI/pDNA polyplexes are generally larger with a higher degree of GA substitution than PPI/pDNA polyplexes (with the exception of GA-PPI-8). This trend was further confirmed by scanning electron microscopy (SEM) and transmission electron microscopy (TEM) images in Fig. S5, showing the smaller GA-PPI-5/pDNA polyplexes with more uniform size distribution (~100 nm) in comparison to PPI/pDNA (200 ~ 400 nm). Figure 2B compares the zeta potential values of the polyplexes, and shows the zeta potential value increases with the N/P ratio and decreases with the GA substitution degree. Except for GA-PPI-7 and GA-PPI-8, the zeta potential remains positive at N/P ratios above 1.0.

The results above suggest the introduction of hydrophilic GA can partially neutralise the high positive charge of PPI dendrimer, leading to more compact structure and better stability when forming polyplexes with negatively charged pDNA. Importantly, the polyplex size and zeta potential can be fine-tuned in a relatively broad range by changing the GA substitution degree and N/P ratio. In summary, the biophysical properties of the modified GA-PPI dendrimers suggest that they are potentially better candidates for gene delivery than existing PPI polyplexes, since smaller size and lower positive charges are favoured by endocytosis mechanisms through negatively charged proteoglycans on cell surfaces, while minimising cell damag^33^,^34^.

### Gene Loading and Protective Ability of GA-PPI polyplexes

Efficient gene loading and the ability to protect encapsulated DNA are desired properties for gene carrier/pDNA polyplexes, as they have to overcome a series of barriers to successfully transport DNA to target cells without being digested by various nucleases in cells or *in vivo*^35^. The gene binding ability of GA-PPI dendrimers with different GA substitution degrees was examined by gel retardation assays using naked pDNA as the polyplex cargo. As shown in Fig. 3A, the electrophoresis mobility of free pDNA decreases as the mixing charge (N/P) ratio increases, such that eventually all the pDNA can be bonded to the polyplex (and accordingly pDNA is completely retarded from migrating through the gel and hence become stuck on the top of the agarose gel) for GA-PPI-1 to -7 when mixing charge (N/P) ratios were above 5.0. By contrast, the gene loading capability of GA-PPI-8 was weak indicating high GA substitution (32.08%) further limits its application as gene carrier. The experimental results suggest that the GA substitution ranging from 0.9% to 23.7% does not significantly affect the gene loading capability of GA-PPI. Next, the protection capability of GA-PPI to nucleic acid against nuclease degradation was evaluated (using pDNA as the cargo nucleic acid). 0.2 μg of naked pDNA was completely degraded after incubation with 200 U/mL of DNase I (an excess of enzyme to DNA) at 37 °C for 30 min (Fig. 3B). However, the pDNA can be fully protected by the GA-PPI polyplexes (1 to 6) at N/P ratios above 3. The GA-PPI-7 and GA-PPI-8 cannot efficiently protect the loaded pDNA, which may due to the fact that high GA substitutions (>23.7%) interfere with pDNA binding (Fig. 3B). Given that nuclease concentration *in vivo* is reported to be 20 times lower than our experimental DNase concentration^36^, we predict that our GA-PPI dendrimers (−1 to −6) represent excellent candidate gene-carriers for gene therapy.

### Cytotoxicity

The cytotoxicity of GA-PPI dendrimers was investigated against a variety of cell types (CHO, HEK 293, MSC, and HepG2) in a broad concentration range (1.0–50.0 μg/mL), with the original PPI dendrimer as the control. Figure 4A summarises the MTT cell viability assay results for CHO cells. The PPI dendrimer was highly toxic, with less than 50% of CHO cells surviving beyond 5.0 μg/mL PPI concentrations. However, GA-PPI-4 to GA-PPI-8 (with GA substitution degree 6.31–32.08%) offer excellent biocompatibility, with cell viabilities over 90% for the entire testing concentration range. Similar results were obtained for the other cell types (Fig. 4B–D), suggesting the cytotoxicity of PPI dendrimer can be removed through controlled GA conjugation. For comparison purpose, the cytotoxicity of GA-PPI/pDNA polyplexes was tested with liver model cell (HepG2) using bPEI/pDNA and PPI (G4)/pDNA as controls. The results demonstrate that the cell viability 48 hours after treatment with GA-PPI (94.3%) is much higher than those of PPI (75.2%) and bPEI 25 K (62.5%) (Fig. S6), indicating that the cytotoxicity of PPI dendrimer is significantly improved after GA coupling, towards excellent biocompatibility. The results above are consistent with the zeta potential measurement, since the high positive charge of the original PPI dendrimer was reported to be the major cause of its high cytotoxicity^10^,^17^. The minimal cytotoxicity of GA-PPI is further confirmed by an acridine orange (AO)/ ethidium bromide (EB) assay. EB is able to penetrate through the cell membranes of normal and necrotic cells, while AO is only taken up by necrotic cells with damaged membranes. Accordingly, orange/green double-labelled cells are necrotic. As shown in Fig. S7, GA-PPI-4 (200 μg/mL) treated HepG2 cells were only observed with green fluorescence, while PPI (G4) and bPEI 25 kD (100 μg/mL) treated cells were observed with both green and red fluorescence, which is consistent with the cytotoxicity data from the MTT assay. To further investigate the cumulative toxicity of GA-PPI/pDNA after gene transfection, HepG2 cells were tested with AO/EB and MTT assay at 24 hrs, 48 hrs and 72 hrs after cell transfection. As demonstrated in Fig. S8, the HepG2 cell was not significantly necrotic in the AO/EB assay, which is consistent with the slight drop of cell viability (from 96.3% to 90.6%) in MTT assay. Those results indicate the negligible cumulative toxicity of GA-PPI. Therefore, GA conjugation is able to efficiently minimize the cytotoxicity of PPI dendrimer via reducing the positive charge when the substitution is above 6.31%, and the higher GA substitution (>6.31%) will make no significant difference.

### Cellular Uptake

To evaluate the targeting capability of our GA-PPI dendrimers as gene carriers, we attempted delivery of YOYO-1 labelled pDNA into cultured cells. The YOYO-1 labelled pDNA was delivered by GA-PPI-4 into non-liver cells (CHO) and typical liver cells (HepG2) at the N/P of 10 using PPI dendrimer as positive controls. To identify the location of YOYO-1 pDNA (green fluorescence), cell membrane and nucleus were stained by Alexa Fluor 594 (red fluorescence) and Hoechst 33258 (blue fluorescence), respectively. The images were captured with a confocal microscopy at 6 h post transfection. As shown in Fig. 5A, the green fluorescence of YOYO-1 pDNA can be detected in cytoplasm of CHO cells after 6 h pDNA delivery both for PPI dendrimer and GA-PPI-4. However, the fluorescent intensity of YOYO-1 pDNA delivered by GA-PPI-4 was much weaker than that of PPI dendrimer. The surface charge density of GA-PPI/pDNA polyplexes significantly decreased after GA conjugation comparing to that of PPI dendrimer, which reduced the probability that the carrier/pDNA polyplexes electrostatically interact with negatively charged proteoglycans of cell membranes and further limits the polyplexes enter into cells through regular endocytosis. Therefore, the GA conjugation leads to low non-specific pDNA deliver capability of GA-PPI dendrimers for non-liver cells. As for the typical liver cells (HepG2), the fluorescence intensity of labelled pDNA delivered by GA-PPI-4 was significantly stronger than that of PPI dendrimer in HepG2 cells (Fig. 5B). GA receptor is over-expressed on the cell membrane of liver cell including HepG2 cell, therefore, GA-PPI dendrimers could deliver pDNA into HepG2 cells *via* an efficient GA receptor-mediated endocytosis pathway instead of normal endocytosis, leading to a high-performance of cellular uptake. On the other hand, the fluorescence intensity of labelled pDNA delivered by PPI dendrimer was similar when evaluated with non-liver cells (CHO) and typical liver cells (HepG2), resulting from the same cell uptake mechanism and pathway. The developed GA-PPI dendrimers have low non-specific capability with non-liver cells, but can efficiently transport therapeutical gene into liver cell. These experimental results indicate the excellent gene targeted delivery capability of GA-PPI dendrimers as targeted gene carriers for liver cells.

### Cell transfection

Considering the gene loading and protection capability, formed particles’ sizes and cytotoxicity, GA-PPI-4 to GA-PPI-6 were eventually selected for the *in vitro* cell transfection experiment using pEGFP-N1 pDNA as model gene. This was again carried out with non-liver cells (CHO) and typical liver cells (HepG2) to verify the targeting specificity, quantified by flow cytometry. As shown in Fig. 6, for non-liver (CHO) cells, PPI was approximately twice as efficient as GA-PPI (highest efficiency ~20% compared with ~10%), and at a fixed N/P ratio, the transfection efficiency of GA-PPI generally decreased with higher GA substitution degree. These results suggest that the higher complexity/size of GA-PPI polyplexes impedes endocytic uptake. For liver (HepG2) cells, the percentage of cells transfected by GA-PPI was significantly higher than that of PPI (Fig. 6B) with highest efficiency ~43% compared to ~15%. This demonstrates efficient GA receptor-mediated gene delivery of GA-PPI dendrimers. In addition, the cell transfection efficiencies of GA-PPI-6 are lower than those of GA-PPI-4 and -5, which indicate that the high GA substitution (above 15.64%) is not necessary. The high targeting capability of GA-PPI dendrimers for liver cells was also confirmed by fluorescent images (Fig. 6C). It is notable that the GA conjugation to PPI dendrimer can improve the biocompatibility and liver cell targeted capability of PPI dendrimer, but partly weaken its gene loading/protection ability and buffering capability (Fig. S9, Supporting Information). Therefore, a balance between gene loading and protection capability, buffer capability, cytotoxicity and liver cells targeted transfection efficiency need to be kept by the adjustment of GA substitution degree. After the GA substitution optimization, GA-PPI-4 was compared with the current gold standard gene carrier, bPEI-25 K, in transfection efficiency of HepG2 liver cells. As can be seen, the transfection efficiency of GA-PPI-4/pDNA is twice higher than that of PEI-25 K/pDNA (43.5% *vs* 22.3%) (Fig. S10). Moreover, HepG2 cells were transfected by GA-PPI-4/pDNA in the presence of various serum concentration (0–50%) to simulate *in vivo* environment, with no obvious difference observed in transfection efficiency (Supplementary Fig. S11A). However, the cell transfection efficiency of bPEI 2 K and PPI significantly decreased with the increment of serum concentration (Fig. S11B). This suggests GA-PPI dendrimers are not affected by serum in the transfection medium (which may be due to their low surface charge after conjugation), and can be potentially applied *in vivo* in complex biological solutions. Therefore, GA-PPI dendrimers represent a potential, efficient gene carrier for liver cells.

## Conclusions

In this study, we successfully developed a new delivery system with good biocompatibility and efficient liver cell targeting capability through one-step GA conjugation to PPI dendrimer (GA-PPI). One should note that GA substitution is the key factor to control the gene loading/protection, cytotoxicity, targeting transfection efficiency of resulted GA-PPI. With optimal substitution (6.31%), GA-PPI demonstrates excellent water solubility, and can efficiently load pDNA and form stable nanostructure with good pDNA protection capability. Furthermore, such GA-PPI dendrimers have low toxicity to different types of cells from various tissues after GA conjugation. Most importantly, GA-PPI dendrimers have highly efficient targeted gene delivery capability for cultured liver cells since the GA on its backbone can trigger GA receptor mediated cellular uptake pathway, which does not affect by the serum and work very well in the mimetic *in vivo* environment. Comparing to gold standard of gene carrier (bPEI 2 K), the developed GA-PPI demonstrates lower cytotoxicity (cell viability, 94.3% *vs* 62.4%) but higher cultured liver cell transfection efficiency (43.5% vs 22.3%) with targeting, which suggest its good potentials as gene carrier. Therefore, we successfully demonstrated the principal of concept on how to develop high-performance gene carriers based on PPI dendrimers via one step conjugation and identified with *in vitro* investigation in this work, the resulted delivery system need to be tested in the animal disease models in the future work before the clinical application.

## Methods

### Materials

Generation 4 diaminobutyric polypropylenimine (PPI) dendrimer, 1-ethyl-3-(3-dimethy- laminopropyl) carbodiimide (EDC) and N-hydroxysulfosuccinimide (NHS) were purchased from Acros (New Jersey, USA). QIAGEN Maxi kit was obtained from Qiagen (Boncaster, Australia). Plasma membrane and nuclear labelling kit, nucleic acid stains dimer sampler were purchased from Life Technologies (Mulgrave, Australia). Fetal bovine serum (FBS), trypsin-EDTA, penicillin-streptomycin (PS) mixture, DMEM cell culture medium, phosphate buffered saline (PBS), tris-acetate (TAE), agarose and Lipofectamin^TM^ 2000 reagent were purchased from Gibco-BRL (Grand Island, USA). Sucrose, gel red, 3-(4, 5-dimethylthiazol-2-yl)-2, 5-diphenyltetrazolium bromide (MTT), kanamycin, glycyrrhetinic acid (GA) and other chemicals/solvents were purchased from Sigma-Aldrich (St. Louis, MO).

### Synthesis of GA-PPI

The synthesis of GA-PPI dendrimer is described in Fig. S1. A serial of GA functionalized PPI dendrimer (GA-PPI) with different GA substitution degree were synthesized and purified. Taking GA-PPI-1 for example, NHS/EDC (3.017 mg/5.023 mg, 0.0064 mmol) and GA (3.008 mg, 0.0064 mmol) were added to 10 mL MES buffer at pH 5.5 and stirred at room temperature for 1 h. It was then mixed with PPI solution (200 mg, 0.64 mmol amine group of PPI) dissolved in 15 mL MES buffer at pH 5.5. The mixture was stirred in darkness at room temperature for 16 h, followed by dialysis against deionized water (pH 7.4) for another 5 days. The obtained GA-PPI dendrimers were lyophilized, and primarily confirmed by the ^1^H-NMR (600 MHz, D_2_O) spectral data : δ 2.40–2.50 (br m, -CH_2_CONH-), δ 2.62–2.73 (br m, -NHCH_2_CH_2_NH-), δ 2.82–2.92 (br m, -NCH_2_CH_2_CONH-), δ 3.06–3.17 (m, CH_2_NHCOCH_2_-), δ 0.64–1.37 ppm (43 H, typical protons of GA moiety).

### Determination of GA substitution degree

Since GA has a specific absorption peaks at 250 nm, a UV-visible spectrophotometer (UV-1601, SHIMADZU) was used to determine the degree of GA substitution along the PPI dendrimer backbone. After the calibration curves were set up at pH 7 (Fig. S2, with path length of 1 cm), the GA substitution degree of the synthesized GA-PPI dendrimers was determined from the absorption peaks at 250 nm according to the Beer-Lambert’s law^37^. Detailed data were concluded in the Supplementary Table S1.

### Size and zeta potential of GA-PPI/pDNA polyplexes

Various polyplexes were prepared by mixing GA-PPI dendrimers with 5.0 μg naked pDNA at different charge (N/P) ratios at pH 7.2 under room temperature for 20 min. The size and zeta potential were measured by a Malvern Zetasizer (Malvern Inst. Ltd. UK) equipped with a four-side clear cuvette or ZET 5104 cell at room temperature^38^. The N/P ratio of the polyplexes was expressed as the molar ratios of the amine groups in (GA-) PPI to the phosphate in pDNA. For the N/P charge ratio calculation, 330 Da was used as the average mass per charge for pDNA, and the average mass per charge for (GA-) PPI was calculated as an average mass per N atom for the whole gene carrier. The cumulant method was used to convert intensity-intensity autocorrelation functions to apparent particle sizes according to the Stokes-Einstein relationship^39^. The Smuloschowski model was used to convert electrophoresis mobility to zeta potential^40^. Ten parallel runs were carried out for each measurement and statistical analysis was applied to the final data.

### Gel electrophoresis

To evaluate the gene loading capacity, the GA-PPI/pDNA polyplexes prepared at different N/P ratios were loaded onto 0.8 wt% agarose gel in a TAE running buffer and electrophoresed at 80 V for 60 min. The resulting pDNA migration patterns were read under UV irradiation (G-BOX, SYNGENE). To evaluate the gene protection capacity, the GA-PPI/pDNA polyplexes were incubated with DNase I (25 μL,160 units/mL) in DNase/Mg^2+^ digestion buffer (50 mM, Tris-HCl, pH 7.6, and 10 mM MgCl_2_) at 37 ^o^C for 30 min, along with free pDNA (0.2 μg) as the negative control. The digestion of pDNA was investigated by 0.8 wt% agarose gel with a TAE running buffer and electrophoresed at 80 V for 60 min. The results were read under UV irradiation^41^.

### Cytotoxicity assay

Normal cell (CHO), mesenchymal stem cells (MSC), human embryonic kidney (HEK293) and liver cancer cell (HepG2) were cultured in DMEM medium supplied with 10% FBS in 96-well plates (200 μL/well) at a cell density of 1.0 × 10^5^ cells/mL. After inoculation, the cells were allowed to adhere overnight at 37 °C in a humidified 5% CO_2_-containing atmosphere. The growth medium was replaced with 200 μL fresh medium containing GA-PPI dendrimer at final concentrations of 0.5, 1, 3, 5, 10, 20, 30, 50 μg/mL. Cells were then incubated for 48 h before 10 μL of MTT (5.0 mg/mL in PBS) was added to each well for the evaluation of cell viability. After incubating for another 4 h at 37 °C, the growth medium was replaced by 150 μL of dimethyl sulfoxide to ensure complete solubilisation of the formed formazan crystals. Finally, the absorbance was determined using the Biotek Microplate Reader (Biotek, USA) at the wavelength of 570 nm^42^,^43^. The cytotoxicities of GA-PPI-4, PPI and bPEI 25 kD were further tested with HepG2 cell using an acridine orange (AO)/ethidium bromide (EB) double-staining experiment. Generally, cells were cultured in a 24-well plate in DMEM for 24 h. The cells were incubated with the tested materials for 12 h and the cells were then washed with PBS and stained by AO and EB containing PBS buffer (5 μg/mL AO and EB) for 10 min. The stained cells were imaged by fluorescence microscope^43^.

### Intracellular uptake

CHO and HepG2 cells at a concentration of 2 × 10^5^ cells/well were cultured in 6-well plates loaded with cover-glass slides for 24 h. 4 μg YOYO-1 labelled pDNA (labelling molar ratio of 1 dye molecule to 100 nucleic acid base pairs) was loaded onto the different gene carriers (PPI, GA-PPI-5) at N/P ratios of 5.0 to form (GA-) PPI/pDNA polyplexes. Cells were incubated with the polyplexes for another 6 h, and then the polyplexes were removed by washing the cells with PBS for three times before fixing with 4% formaldehyde. The cell membranes and nuclei were separately stained by 100 μL of Alexa Fluor 594 (5.0 μg/mL) and Hoechst 33258 (2 μM) for 15 min at 37 °C. The cells were further washed with PBS for three times, and incubated with 500 μL PBS at room temperature for further analysis. The fluorescent images were observed by a confocal laser scanning microscope (Leica Confocal 1P/FCS) equipped with a 405 nm diode laser for Hoechst 33258, a 488 nm argon ion laser for YOYO-1 and a 561 diode laser for Alexa Fluor 594. The high magnification images were obtained with a 100 × objective, and averaged for 4 times to reduce noise. The images were processed using the Leica Confocal software^44^.

### Cell transfection experiment

The pEGFP-N1 plasmid expressing the Enhanced Green Fluorescent Protein (EGFP) was prepared in *E*. *coli* DH5α strain and extracted using a QIAGEN Maxi kit. The integrity and purity of the prepared plasmid DNA was analysed using 0.8% agarose gel electrophoresis and the DNA concentration was determined using a Jasco UV-vis spectrophotometer (Tokyo, Japan) at the fixed wavelengths of 260 and 280 nm^45^.

CHO and HepG2 cells were seeded in 24-well plates and cultured in complete DMEM supplemented with 10% fetal bovine serum (FBS) at 37 °C in a humidified incubator, in the presence of 5% CO_2_. After 24 h culturing, the medium was replaced with 200 μL fresh culture medium in the absence of FBS. The as-prepared polyplexes were then added to each well. After 6 h incubation, the cultured medium was replaced with 1 mL fresh culture medium with 10% FBS, and the cells were further incubated for another 42 h.

To quantify the transfection efficiency, the cells were harvested by the trypsin digestion method after 42 h post-transfection. 1 × 10^6^ cells were obtained and washed with 2% FCS/PBS buffer, and centrifuged at 1000 rpm for 5 min. The cells were stained by propidium iodide (PI, 400 μL, 0.5 μg/mL) in 1 × PBS to select the live cells. A FACS Calibur flow cytometry (Becton Dickinson) was used to count the number of transfected cells by detecting the green fluorescence of EGFP with non-transfection cells (mock cells) as the negative control. Approximately 1–2 × 10^4^ cells were analysed at the rate of 200 ~ 600 cells per second. CellQuest3.3 software was used for data analysis, and the transfection efficiency was calculated as the percentage of positive cells to total cells. The EGFP GFP expression was also verified by fluorescence microscopy. Briefly, the post-transfection living cells were rinsed 3 times by 1 × PBS and visualized *in situ* under an epi-fluorescence microscope (Multi-photon Microscope, Nikon) with a band pass excitation filter (BP 485/20) and a 520 nm long-pass emission filter. Digital images were captured by a CCD camera (RS Photometrics), and analysed using the Bio-Rad Radiance 2000 MP Visualising System^46^.

### Statistical Analysis

The experimental data of all variables were analysed using a two-sample, two-tailed t-test, and the results were represented as mean ± SE (standard error).

## Additional Information

**How to cite this article**: Cong, Y. *et al.* One-step Conjugation of Glycyrrhetinic Acid to Cationic Polymers for High-performance Gene Delivery to Cultured Liver Cell. *Sci. Rep.* **6**, 21891; doi: 10.1038/srep21891 (2016).

## Supplementary Material

Supplementary Information

## Figures and Tables

**Figure 1:** Scheme for the targeted gene delivery of GA equipped PPI dendrimers (GA-PPI). After GA conjugation, the GA-PPI derivatives can efficiently load therapeutic gene and form nanostructures polyplexes via self-assembling. The resulted polyplexes is able to specifically deliver therapeutic genes into liver cells with negligible cytotoxicity.

**Figure 2:** Particles size (**A**) and zeta-potentials (**B**) of the GA-PPI/pDNA polyplexes prepared at eight different mixing charge (N/P) ratios of polymer to pDNA at pH 7.2, 25 °C. For all measurements, the DNA concentration was fixed at 5 μg/mL. The size and zeta potential were measured by a Malvern Zetasizer (Malvern Inst. Ltd. UK) equipped with a four-side clear cuvette or ZET 5104 cell at room temperature. The N/P ratios of the polyplexes were expressed as the molar ratios of the amine groups in (GA-) PPI to the phosphate in pDNA (Calculation details, see Method section).

**Figure 3:** Nucleic acid binding and protection ability assay of GA-PPI dendrimers by agarose gel electrophoresis using 0.8% agarose in Tris-acetate running buffer. (**A**) Nucleic acid binding ability assay; (**B**) Nucleic acid protection capability assay against DNase І. The GA-PPI/pDNA (pEGFP-N1: 4.7 kb) polyplexes were prepared at various mixing charge (N/P) ratios with fixed amount of pDNA (0.2 μg) at pH 7.2. The GA-PPI/pDNA polyplexes were loaded on the agarose gel and analyzed with gel electrophoresis system directly for nucleic acid binding capability assay. As for DNA protection ability assay, GA-PPI/pDNA polyplex and free pDNA (0.2 μg) were separately incubated with DNase I (4 units) in DNase/Mg^2+^ digestion buffer (50 mM, Tris-Cl, pH 7.6, and 10 mM MgCl_2_) at 37 °C for 30 min and the degradation of pDNA was investigated by 0.8% agarose gel electrophoresis.

**Figure 4:** Comparison of the cytotoxicity of the synthesized GA-PPI dendrimer carriers, PPI dendrimer against various cell lines using unmodified PPI as control. (**A**) CHO cells; (**B**) MSC cells; (**C**) HEK 293 cells; (**D**) HepG2 cells. The absorbance was read at 570 nm using a microplate reader (n = 3). For all the cell lines from different tissue sources, the cytotoxicity of PPI was significantly improved after GA conjugation, the higher substitution degree, the less cytotoxicity of GA-PPI.

**Figure 5:** Comparison of cellular uptake of YOYO-1-labeled pDNA delivered by GA-PPI dendrimer and PPI dendrimer with various types of cells. (**A**) CHO cells; (**B**) HepG2 cells. Cells were visualized using a confocal 1P/FCS inverted microscope after cell membrane and nucleus were stained with 100 μL of Alexa Fluor 594 (5.0 μg/mL) and Hoechst 33258 (2 μM). Both PPI and GA-PPI-4 were poor delivery vehicles for CHO cells, with low levels of detection of YOYO-1 labelled DNA inside cells. However, GA-PPI-4 can very effectively deliver YOYO-1 labelled DNA into HepG2 cells comparing to PPI dendrimers.

**Figure 6:** Cell transfection capability of GA-PPI/pDNA polyplexes were evaluated with normal cell (using CHO as a model cell line) and liver cell (using HepG2 as a model cell line) at various mixing charge ratios with positive control PPI dendrimer. (**A**) CHO cells; (**B**) HepG2 cells. Transfection efficiencies were determined by flow cytometer and cell images were captured with fluorescent microscopy, data shown as mean ± SE (n = 3).
